The article "Exosomal DLX6-AS1 from hepatocellular carcinoma cells induces M2 macrophage polarization to promote migration and invasion in hepatocellular carcinoma through microRNA-15a-5p/CXCL17 axis" was retracted in 2022. Reasons: original data or images not available; unreliable results or conclusions; concerns about the images.

# Exosomal DLX6-AS1 from hepatocellular carcinoma cells induces M2 macrophage polarization to promote migration and invasion in hepatocellular carcinoma through microRNA-15a-5p/CXCL17 axis

**DOI:** 10.1186/s13046-021-01973-z

**Published:** 2021-05-26

**Authors:** Lin-pei Wang, Jing Lin, Xiao-qiu Ma, Dong-yao Xu, Chun-feng Shi, Wei Wang, Xiao-jie Jiang

**Affiliations:** 1 Department of Hepatobiliary and Pancreatic Surgery, The Second Affiliated Hospital of Fujian Medical University, Quanzhou, 362000 Fujian China; 2 Department of Pathology, Affiliated Putian Hospital of Putian College, Putian, 363100 Fujian China; 3 Department of Internal Medical Oncology, The 910th Hospital of the People’s Liberation Army, Quanzhou, 362000 Fujian China; 4 Department of Hepatobiliary Surgery, Affiliated Putian Hospital of Putian College, Putian, 363100 Fujian China

**Keywords:** Hepatocellular carcinoma, Hepatocellular carcinoma cell-secreted exosomes, M2 macrophages, Long non-coding RNA distal-less homeobox 6 antisense 1, microRNA-15a-5p, C-X-C motif chemokine ligand 17

## Abstract

**Background:**

Hepatocellular carcinoma (HCC) cells-secreted exosomes (exo) could stimulate M2 macrophage polarization and promote HCC progression, but the related mechanism of long non-coding RNA distal-less homeobox 6 antisense 1 (DLX6-AS1) with HCC-exo-mediated M2 macrophage polarization is largely ambiguous. Thereafter, this research was started to unearth the role of DLX6-AS1 in HCC-exo in HCC through M2 macrophage polarization and microRNA (miR)-15a-5p/C-X-C motif chemokine ligand 17 (CXCL17) axis.

**Methods:**

DLX6-AS1, miR-15a-5p and CXCL17 expression in HCC tissues and cells were tested. Exosomes were isolated from HCC cells with overexpressed DLX6-AS1 and co-cultured with M2 macrophages. MiR-15a-5p/CXCL17 down-regulation assays were performed in macrophages. The treated M2 macrophages were co-cultured with HCC cells, after which cell migration, invasion and epithelial mesenchymal transition were examined. The targeting relationships between DLX6-AS1 and miR-15a-5p, and between miR-15a-5p and CXCL17 were explored. In vivo experiment was conducted to detect the effect of exosomal DLX6-AS1-induced M2 macrophage polarization on HCC metastasis.

**Results:**

Promoted DLX6-AS1 and CXCL17 and reduced miR-15a-5p exhibited in HCC. HCC-exo induced M2 macrophage polarization to accelerate migration, invasion and epithelial mesenchymal transition in HCC, which was further enhanced by up-regulated DLX6-AS1 but impaired by silenced DLX6-AS1. Inhibition of miR-15a-5p promoted M2 macrophage polarization to stimulate the invasion and metastasis of HCC while that of CXCL17 had the opposite effects. DLX6-AS1 mediated miR-15a-5p to target CXCL17. DLX6-AS1 from HCC-exo promoted metastasis in the lung by inducing M2 macrophage polarization in vivo.

**Conclusion:**

DLX6-AS1 from HCC-exo regulates CXCL17 by competitively binding to miR-15a-5p to induce M2 macrophage polarization, thus promoting HCC migration, invasion and EMT.

**Supplementary Information:**

The online version contains supplementary material available at 10.1186/s13046-021-01973-z.

## Background

Liver cancer is a morphologically heterogeneous tumor with variable structural growth patterns and different histological subtypes [1]. Continued increases of hepatocellular carcinoma (HCC) mortality until 2030 has been predicted [2]. Miserably, early diagnosis for liver cancer is rare due to the vague symptoms and the lack of effective identification and screening [3]. Liver transplantation, local ablation, surgical resection, systemic therapy with tyrosine kinase inhibitors and transarterial chemoembolization have been introduced to liver cancer treatment [3]. However, there still are concerns in managing liver cancer, such as unexpected progression-free survival, drug resistance and relapse [4]. In such a predicament, exploring effective agents to treat liver cancer is the prior task.

Macrophage polarization is related to tumorigenesis and M2 macrophages support tumor growth [5]. Tumor-associated macrophages (TAMs) have been established to act as a driving factor for M2 macrophages, leading to tumor growth, invasion and metastasis [6]. Tumor-derived exosomes can be ingested by macrophages in the tumor microenvironment and ultimately promote tumor progression and metastasis [7]. HCC-derived exosomes (HCC-exo) have been noted to induce M2 macrophages [8, 9]. Long non-coding RNA (lncRNA) TUC339 derived from HCC-exo has been implied to regulate macrophage activation and polarization [10], suggesting the interaction of tumor exosomal lncRNAs and macrophage polarization in cancer development. LncRNA distal-less homeobox 6 antisense 1 (DLX6-AS1) is a prognostic biomarker in liver cancer [11], whose down-regulation impairs the stemness of cancer cells [12]. Moreover, silenced DLX6-AS1 serves satisfactorily for suppressing the biological functions of HCC cells [13]. MicroRNAs (miRNAs) are also of great importance in liver cancer such as miR-15a-5p. Actually, enhanced level of miR-15a-5p could block liver cancer cell proliferative activity, as well as other pro-tumorigenic activities [14, 15]. miR-15a-5p has been testified to target C-X-C motif chemokine ligand 10 (CXCL10) to suppress metastasis in chronic myeloid leukemia [16], implying the potential mechanism of miR-15a-5p with CXCL in cancers. Belonging to CXCL family, CXCL17 has been implicated to link with prognosis and immune infiltration in HCC [17]. It has been witnessed that highly expressed CXCL17 elicits the malignant phenotypes of liver cancer cells [18]. In our study case, we aimed to figure out whether tumor cells-derived exosomal DLX6-AS1 could interact with miR-15a-5p/CXCL17 axis in HCC metastasis through polarizing M2 macrophages.

## Methods

### Ethics statement

All patients signed an informed consent form. The study was approved by the Ethics Committee of Affiliated Putian Hospital of Putian College. All animal experiments were approved by the Institutional Animal Care and Use Committee.

### Experimental subjects

Cancer tissues and normal tissues (76 pairs) were collected. Normal tissues were resected at least 3 cm from the tumor. None of the patients received chemotherapy or radiotherapy before surgery. All tissues were immediately frozen in liquid nitrogen and preserved at − 80 °C [19].

### Immunohistochemical staining

HCC tissue samples were fixed with 4% neutral paraformaldehyde buffer (p1110, Solarbio, Beijing, China), embedded in paraffin and sectioned continuously with a thickness of 4 μm. The slices were baked at 60 °C for 1 h, dewaxed and hydrated in xylene I and xylene II, dehydrated with gradient alcohol, and soaked in 3% hydrogen peroxide for 20 min to eliminate the activity of endogenous peroxidase. Then, the slices were washed with phosphate buffer (PBS), sealed with 10% goat serum for 15 min and incubated with primary antibody CD68 (1: 150, ab201973, Abcam, MA, USA) overnight at 4 °C, and then were washed with PBS for three times, incubated with biotinylated goat anti-rabbit immunoglobulin G (IgG, ab97051, 1: 2000, Abcam) second antibody working solution for 40 min and developed by diaminobenzidine (DAB, da1010, Solarbio) for 10 min. Subsequently, the slices were counterstained with hematoxylin (h8070, Solarbio) for 1 min, washed with running water, dehydrated with gradient ethanol, permeabilized using xylene and sealed with neutral gum. PBS was used as negative control (NC) instead of primary antibody. Finally, five high-power fields were randomly selected under the light microscope (cx41-12c02, Olympus, Tokyo, Japan) and the results were scored using double-blind method. The brown yellow particles in the cells were regarded as the positive cells, which were calculated according to the percentage of the total cells.

### Cell culture

Human HCC cell lines (SMMC-7721 and HepG2), human normal hepatocytes HL-7702, and monocyte cell line THP-1 (American Type Culture Collection, VA, USA) were kept in Dulbecco’s Modified Eagle Medium (DMEM) plus 10% fetal bovine serum (both from Thermo Fisher Scientific, MA, USA). THP-1 cells (1 × 10^6^) were induced by 100 ng/mL phorbol 12-myristate 13-acetate (PMA, Sigma-Aldrich, SF, USA) for 24–48 h [19].

### Isolation and identification of exosomes

SMMC-7721 cells were cultivated to 80–90% confluence and 3 d later, the culture medium (30 mL) was centrifuged (300 g, 2000 g, 10,000 g and 100,000 g) to collect the pellet which was then resuspended in 50–100 μL PBS [20]. As previously described [21], Exoquick-TC™ kits (EXOTC50A-1, Systembio, CA, USA) were used to isolate the exosomes through precipitation method. In brief, the resuspension was incubated with Exoquick reagent (5:1) for more than 12 h, centrifuged at 1500 g, resuspended in PBS (100 μL) and placed at − 80 °C. In addition, serum exosomes were isolated by total exosomes separation reagent (Magen, NY, USA). The serum (1 mL) was mixed with the exosomes separation reagent, centrifuged at 2000 g and 10,000 g and resuspended in 200 μL PBS. Exosomes were suspended in glutaraldehyde, dropped into a carbon-coated copper grid, stained with 2% uranyl acetate and examined by transmission electron microscopy.

### Exosome labeling

The purified exosomes isolated from the culture medium were labeled with PKH67 fluorescence (Sigma), resuspended and added to macrophages. The exosomes were suspended in 1 mL Diluent C solution, which was added with 4 μL PKH26 ethanol dye solution to prepare 4 × 10^− 6^ M dye solution. The exosome suspension (1 mL) was mixed with dye solution for 5 min and the staining was stopped through the 1-min incubation with 2 mL 1% exosome-depleted fetal bovine serum (FBS). The labeled exosomes were ultracentrifuged at 100,000×g for 2 h to enrich the exosomes in the range of 1.13–1.19 g/ml sucrose density [22]. Then, the labeled exosome sediment was resuspended and added into the unstained macrophages for the exosome uptake experiment. Cells were incubated for 30 min, 2 h or 12 h, and then were observed under a fluorescence microscope [21].

### Cell transfection

Lentiviral vector construction and cell transfection were performed as previously described [19]. Briefly, cDNA encoding DLX6-AS1 was amplified by Pfu Ultra II Fusion HS DNA polymerase (Stratagene, Agilent Technologies, CA, USA) and cloned into pSin-EF2-Sox2-Pur (Addgene, MA, USA). Oligonucleotides and corresponding negative controls (NCs) that overexpressed or lowly-expressed DLX6-AS1 (RiboBio, Guangzhou, China) were cloned into the lentiviral expression vector pLKO.1-Pur (Addgene). According to the manufacture’s protocol, 293 T cells were incubated with the mentioned vectors for 24 h, and the supernatant containing lentivirus was filtered using a 0.22 μm polyvinylidene fluoride (PVDF) and added onto the plates to transfect the SMMC-7721 and HepG2 cells. The cells were screened with 10 μg/mL puromycin for 4 w and the transfection efficiency was verified using RT-qPCR [19].

Macrophages were performed with transient transfection. The small interfering RNA (si)-CXCL17, miR-15a-5p inhibitor and the relative NCs were purchased from Genechem Co., Ltd. (Shanghai, China). The macrophages were seeded onto the 6-well plates at a density of 4 × 10^5^ cells/mL and cultured, and when the cell confluence reached 80%, the cells were transfected based on instructions of the lipofectamine 2000 reagent (11668–019, Invitrogen, CA, USA). After the transfection, cells were cultured for 48 h and used for the subsequent experiments.

### Flow cytometry

The macrophages were washed with cold PBS and separated with 5 mM ethylene diamine tetraacetic acid. Then, the macrophages (0.5 × 10^6^) were resuspended in 1 mL PBS, added with fluorescein isothiocyanate, phycoerythrin and allophycocyanin conjugated Abs anti-human CD206 (BD Pharmingen, USA). FACScalibur (Beckman Coulter, USA) was used for flow cytometry analysis.

### RNA immunoprecipitation (RIP) assay

Magna RNA-binding protein immunoprecipitation kit (Millipore, MA, USA) was used for detection according to the instructions. In brief, RIP buffer containing magnetic beads conjugated with human anti-Ago2 antibody or NC mouse IgG were added into the cell lysate and incubated with proteinase K. Then, the immunoprecipitated RNA was isolated, with the concentration (a spectrophotometer [Thermo Scientific, MA, USA]) and quality (a bio-analyzer [Agilent]) was evaluated. Finally, RNA was extracted and the purified RNA was detected using RT-qPCR to identify the existence of binding targets [23].

### RNA pull-down assay

Macrophages were transfected with biotinylated wild type (WT) and mutant type (MUT) DLX6-AS1 (50 nm each) for 48 h, and then the cells were collected and incubated with specific cell lysates (Ambion, Texas, USA) for 10 min. After that, 50 mL cell lysate sample was subpackaged and the residual lysates were incubated with M-280 streptavidin magnetic beads (Sigma) precoated with Rnase-free and yeast tRNA (Sigma). Incubated at 4 °C for 3 h, the beads were then washed twice with cold lysate, three times with low salt buffer, and once with high salt buffer. RNA was extracted and detected by RT-qPCR [24, 25].

### Transwell assay

Transwell chamber (Corning USA) contained 24 wells with membrane (8.0 μm). Cells (1 × 10^5^ cells/well) in serum-free medium (100 μL) in the upper chamber were chemo-attracted by the complete medium (600 μL) in the lower chamber. Followed by 24-h incubation, cells in the upper chamber were removed and those in the low chamber were fixed with 4% paraformaldehyde, stained with 0.1% crystal violet solution and photographed by an inverted fluorescence microscope. A total of 100 μL Matrigel (BD, USA) that diluted with DMEM at 1:8 was included in invasion assay [26].

### RT-qPCR

Total RNA Miniprep kit (Axygen, CA, USA) was employed in total RNA extraction from cells and the ReverTra Ace system (Toyobo, Tokyo, Japan) was used in complementary DNA synthesis from RNA (1 μg). Amplification was carried out by Applied Bioscience 7500 system. Table 1 listed the primers.

**Table 1:** Primer sequences

Genes	Primer sequences
DLX6-AS1	F: 5′-AGTTTCTCTCTAGATTGCCTT-3′
	R: 5′-ATTGACATGTTAGTGCCCTT-3′
miR-15a-5p	F: 5′- UUCUCCGAACGUGUCACGUTT-3′
	R: 5′-ACGUGACACGUUCGGAGAATT-3′
CXCL17	F: 5′-ACCGAGGCCAGGCTTCTA-3′
	R: 5′-GGCTCTCAGGAACCAATCTTT-3′
U6	F: 5′-ATTGGAACGATACAGAGAAGATT-3′
	R: 5′-GGAACGCTTCACGAATTTG-3′
GAPDH	F: 5′-ACGGCAAGTTCAACGGCACAG-3′
	R: 5′-GACGCCAGTAGACTCCACGACA-3′
CD206	F: 5′-GGGTTGCTATCAC TCTCTATGC-3′
	R: 5′-TTTCTTGTCTGTTGCCGTAGTT-3′
CD163	F: 5′-ACATAGATCATGCATCTGTCATTTG-3’
	R: 5′-CATTCTCCTTGGAATCTCACTTCTA-3’
CCL17	F: 5′-CAGGAAGTTGGTGAGCTGGTA-3’
	R: 5′-TTGTGTTCGCCTGTAGTGCATA-3’
CCL18	F: 5′-TGGCAGATTCCACAAAAGTTCA-3’
	R: 5′-GGATGACACCTGGCTTGGG-3’

*DLX6-AS1* long non-coding RNA distal-less homeobox 6 antisense 1, *miR-15a-5p* microRNA-15a-5p, *CXCL17* C-X-C motif chemokine ligand 17, *GAPDH* glyceraldehyde-3-phosphate dehydrogenase, *CCL* C-C motif chemokine ligand

### Western blot assay

Radio-immunoprecipitation assay buffer (SenBeiJia Biological Technology Co., Ltd., Nanjing, China) was applied to collect total protein from tissues and cells. The protein concentration was measured bicinchoninic acid protein assay kit (Beyotime, China). About 40 μg of protein was separated by sodium dodecyl sulphate polyacrylamide gel electrophoresis, electro-blotted onto PVDF membrane (Millipore, USA) and blocked with 5% skimmed milk. Antibodies were showed as follows: anti-CXCL17 (AF4207, 1:1000) from R&D Systems (MN, USA), CD63 (sc-5275, 1:1000) and TSG101 (sc-7964, 1:1000) from Santa Cruz Biotechnology (CA, USA), Alix (2171, 1:1000) from Cell Signaling Technology (MA, USA), and horseradish peroxidase-conjugated secondary antibody (1:10,000). The protein expression was detected by Quantity-one software (Bio-Rad Laboratories, USA) with enhanced chemiluminescence kit [26].

### In vivo tumor metastasis assay

Male BALB/c nude mice (4 weeks old; Institute of Zoology, Chinese Academy of Sciences, Beijing, China) were kept in a pathogen-free environment. Mice (*n* = 24/4) were injected with SMMC-7721 cells, as well as HCC-exo-induced macrophages, or macrophages induced by HCC-exo that had been transfected with overexpression (oe)-NC/oe-DLX6-AS1 [21]. SMMC-7721 cells (1 × 10^6^) in 10 μL PBS and macrophages were injected into the right liver lobe in situ. After 3 w, the mice were euthanized, the lungs were collected and fixed with Bouin’s solution to count the number of metastatic lung nodules, and then the lungs were embedded in paraffin for H&E staining.

### Statistical analysis

SPSS13.0 (SPSS, USA) was implicated for data analysis. The data were expressed as mean ± standard deviation. The comparison between two groups was subjected to independent sample t test, while that among multiple groups to One-Way analysis of variance (ANOVA) and Tukey’s multiple comparisons test. *P* < 0.05 was defined as a significant difference.

## Results

### HCC-exo induce M2 macrophage polarization

Exosomes were isolated from SMMC-7721 cells by centrifugation. Observed by electron microscopy, HCC-exo were round with a diameter of about 40–140 nm (Fig. 1a). The HCC-exo markers [27, 28] CD63, Alix and TSG101 (Fig. 1b) were identified using Western blotting, indicating the successful isolation of HCC-exo. Subsequently, THP-1 cells were differentiated into macrophages through PMA, and PMA-induced macrophages grew from a single round suspended cells into adherence, with transparent cytoplasm and strong refractive index (Fig. 1c). Next, the effect of HCC-exo on the polarization of macrophages was uncovered. HCC-exo were labeled by PKH26 and internalized by macrophages (Fig. 1d). M2 macrophage markers [29–31] CD206, CD163, CCL17 and CCL18 were investigated to increase while M1 macrophage markers tumor necrosis factor-α (TNF-α), interleukin (IL)-6 and transforming growth factor β (TGF-β) did not change after co-culture with HCC-exo (Fig. 1e,f). Flow cytometry found that CD206, a marker on the surface of M2 macrophages increased (Supplementary Figure), indicating that HCC-exo induced the polarization of M2 macrophages.

**Fig. 1:** HCC-exo induce macrophage M2 polarization. **a**. Electron microscope observation of the morphology of SMMC-7721 cells-derived exosomes; **b**. Western blot analysis of antigens (CD63, Alix and TSG101) in SMMC-7721 cells-derived exosomes; **c**. Microscopic observation of THP1 cells before and after PMA induction; **d**. PKH26 labeling of exosomes; **e**. RT-qPCR detection of M2 macrophages markers (CD206, CD163, CCL17 and CCL18) after co-culture with HCC-exo; **f**. RT-qPCR detection of M1 macrophages markers (TNF-α, IL-6 and TGF-β) after co-culture with HCC-exo; data were expressed as mean ± standard deviation (repetition = 3) and evaluated by One-way AVONA and Tukey’s test. & *P* < 0.05 compared with the PBS group

### HCC-exo promote migration, invasion and epithelial mesenchymal transition (EMT) via inducing M2 macrophage polarization in HCC

M2 macrophages could promote tumor growth [32]. The effect of HCC-exo-treated M2 macrophages on HCC cell migration, invasion and EMT was determined. HCC-exo-treated M2 macrophages were co-cultured with SMMC-7721 and HepG2 cells, after which cell migration and invasion abilities were enhanced (Fig. 2a,b). Meanwhile, EMT after the co-culture of HCC cells and M2 macrophages was monitored. As analyzed using RT-qPCR, epithelial cell marker E-cadherin expression was decreased, and mesenchymal cell markers (N-cadherin, vimentin, and MMP7 expression) were increased in cells (Figs. 2c). In summary, HCC-exo-treated M2 macrophages promoted migration, invasion and EMT in HCC.

**Fig. 2:** HCC-exo promote migration, invasion and EMT via inducing M2 macrophage polarization in HCC. **a**. Transwell assay tested the invasion and migration of SMMC-7721 cells after co-culture with HCC-exo-treated macrophages; **b**. Transwell assay tested the invasion and migration of HepG2 cells after co-culture with HCC-exo-treated macrophages; **c**. RT-qPCR analysis of E-cadherin, N-cadherin, vimentin and MMP7 mRNA expression in SMMC-7721 and HepG2 cells after co-culture with HCC-exo-treated macrophages; data were expressed as mean ± standard deviation (repetition = 3) and evaluated by One-way AVONA and Tukey’s test. * *P* < 0.05 compared with the SMMC-7721 + M group; ^ *P* < 0.05 compared with the HepG2 + M group

### DLX6-AS1 is overexpressed in HCC and triggers migration, invasion and EMT in HCC

Highly expressed DLX6-AS1 in HCC could promote tumor growth [33]. When investigating the mechanism of DLX6-AS1 in migration, invasion and EMT, DLX6-AS1 expression was firstly tested in cancer tissues and cell lines. It turned out that DLX6-AS1 was up-regulated in cancer tissues and SMMC-7721 and HepG2 cells (Fig. 3a). Subsequently, overexpressed DLX6-AS1 was introduced to SMMC-7721 and HepG2 cells (Fig. 3b). In response to DLX6-AS1 overexpression, SMMC-7721 and HepG2 cells migrated and invaded aggressively (Fig. 3c,d) and EMT [34, 35] was accelerated (Fig. 3e). It was hinted that overexpressed DLX6-AS1 promoted migration, invasion and EMT in HCC.

**Fig. 3:** DLX6-AS1 is overexpressed and triggers migration, invasion and EMT in HCC. **a**. RT-qPCR detection of DLX6-AS1 expression in cancer tissues and normal tissues, as well as cancer cells and normal liver cells; **b**. RT-qPCR detection of DLX6-AS1 expression in SMMC-7721 and HepG2 cells after up-regulating DLX6-AS1; **c**. Transwell assay tested the invasion and migration of SMMC-7721 cells after up-regulating DLX6-AS1; **d**. Transwell assay tested the invasion and migration of HepG2 cells after up-regulating DLX6-AS1; **e**. RT-qPCR analysis of E-cadherin, N-cadherin, vimentin and MMP7 mRNA expression in SMMC-7721 and HepG2 cells after up-regulating DLX6-AS1; data were expressed as mean ± standard deviation (repetition = 3) and evaluated by One-way AVONA and Tukey’s test. $ *P* < 0.05 compared with the HL-7702 cells; * *P* < 0.05 compared with the oe-NC group

### DLX6-AS1 from HCC-exo stimulates M2 macrophage polarization to accelerate migration, invasion and EMT in HCC

Next, to inspect whether DLX6-AS1 was involved in the process of HCC-exo-induced M2 polarization in HCC, DLX6-AS1 expression was examined in exosomes isolated from the serum of HCC patients and healthy controls. As revealed, DLX6-AS1 level was elevated in serum exosome from HCC patients (Fig. 4a). Meanwhile, we detected the distribution of macrophages in HCC tumor microenvironment and analyzed the expression of macrophage marker CD68 in human HCC tissues using immunohistochemical staining. We found that the density of TAMs in cancer tissues was higher than that in adjacent tissues, and it was positively correlated with the expression of exosomal DLX6-AS1 from serum of HCC patients (Fig. 4b, c). Subsequently, DLX6-AS1 level in HCC-exo that had been treated with oe-DLX6-AS1, sh-DLX6-AS1 or the NC was measured. As expected, its expression raised in HCC-exo carrying oe-DLX6-AS1 or decreased in HCC-exo carrying sh-DLX6-AS1 (Fig. 4d, 5a). Next, HCC-exo delivering oe-DLX6-AS1 or sh-DLX6-AS1 were co-cultured with macrophages and the results disclosed that DLX6-AS1 level was increased or decreased in macrophages in a time-dependent manner (Fig. 4e, 5b), confirming that HCC-exo could deliver DLX6-AS1 to macrophages. Next, the role of HCC-exo-delivered DLX6-AS1 in the polarization of M2 macrophages was clarified. After co-culture with HCC-exo-delivered oe-DLX6-AS1 or sh-DLX6-AS1, M2 macrophages markers CD206, CD163, CCL17 and CCL18 were all increased or decreased while no change was observed in M1 markers TNF-α, IL-6 and TGF-β (Fig. 4f, g; 5c, d; Supplementary Figure). Moreover, M2 macrophages treated with HCC-exo transferring oe-DLX6-AS1 were co-cultured with SMMC-7721 and HepG2 cells and then functioned to stimulate cell migration, invasion and EMT. On the contrary, M2 macrophages treated with HCC-exo transferring sh-DLX6-AS1 caused the opposite effect on SMMC-7721 and HepG2 cells (Figs. 4h-j; 5e-h).

**Fig. 4:** DLX6-AS1 from HCC-exo stimulates M2 macrophage polarization to accelerate migration, invasion and EMT in HCC. **a**. RT-qPCR detection of DLX6-AS1 expression in serum of HCC patients and healthy controls; **b**. Detection of CD68 expression in clinical samples through immunohistochemical staining; **c**. Correlation between expression of DLX6-AS1 and CD68 was analyzed using Pearson test; **d**. RT-qPCR detection of DLX6-AS1 expression in HCC-exo delivering oe-DLX6-AS1; **e**. RT-qPCR detection of DLX6-AS1 expression in macrophages after co-culture with HCC-exo delivering oe-DLX6-AS1; **f**. RT-qPCR detection of M2 macrophages markers (CD206, CD163, CCL17 and CCL18) after co-culture with HCC-exo carrying oe-DLX6-AS1; **g**. RT-qPCR detection of M1 macrophages markers (TNF-α, IL-6 and TGF-β) after co-culture with HCC-exo carrying oe-DLX6-AS1; **h**. Transwell assay tested the migration and invasion of SMMC-7721 cells after co-culture with M2 macrophages induced by HCC-exo carrying oe-DLX6-AS1; **i**. Transwell assay tested the migration and invasion of HepG2 cells after co-culture with M2 macrophages induced by HCC-exo delivering oe-DLX6-AS1; **j**. RT-qPCR of E-cadherin, N-cadherin, vimentin and MMP7 mRNA expression in SMMC-7721 and HepG2 cells after co-culture with M2 macrophages induced by HCC-exo delivering oe-DLX6-AS1; data were expressed as mean ± standard deviation (repetition = 3) and evaluated by One-way AVONA and Tukey’s test. * *P* < 0.05 compared with the oe-NC group; # *P* < 0.05 compared with the PBS group; & *P* < 0.05 compared with the oe-NC-exo group; ^ *P* < 0.05 compared with the oe-NC-exo + M group

**Fig. 5:** DLX6-AS1 from HCC-exo stimulates M2 macrophage polarization to accelerate migration, invasion and EMT in HCC. **a**. RT-qPCR detection of DLX6-AS1 expression in HCC-exo delivering sh-DLX6-AS1; **b**. RT-qPCR detection of DLX6-AS1 expression in macrophages after co-culture with HCC-exo delivering sh-DLX6-AS1; **c**. RT-qPCR detection of M2 macrophages markers (CD206, CD163, CCL17 and CCL18) after co-culture with HCC-exo carrying sh-DLX6-AS1; **d**. RT-qPCR detection of M1 macrophages markers (TNF-α, IL-6 and TGF-β) after co-culture with HCC-exo carrying sh-DLX6-AS1; **e**. Transwell assay tested the migration and invasion of SMMC-7721 cells after co-culture with M2 macrophages induced by HCC-exo carrying sh-DLX6-AS1; **f**. Transwell assay tested the migration and invasion of HepG2 cells after co-culture with M2 macrophages induced by HCC-exo delivering sh-DLX6-AS1; **g/h**. RT-qPCR of E-cadherin, N-cadherin, vimentin and MMP7 mRNA expression in SMMC-7721 and HepG2 cells after co-culture with M2 macrophages induced by HCC-exo delivering sh-DLX6-AS1; data were expressed as mean ± standard deviation (repetition = 3) and evaluated by One-way AVONA and Tukey’s test. ^*P* < 0.05 compared with the sh-NC group; *P < 0.05 compared with the oe-NC-exo group; + *P* < 0.05 compared with the oe-NC-exo + M group

### DLX6-AS1 interacts with miR-15a-5p

Then, the potential mechanism of HCC-exo DLX6-AS1 in M2 macrophage polarization, cancer cell invasion, metastasis and EMT was further explored. miR-15a-5p was a new cancer marker that was down-regulated in many cancers and could inhibit HCC development [14, 36]. miR-15a-5p level was detected to be down-regulated in cancer tissues and cell lines (Fig. 6a, b). After that, miR-15a-5p expression was suppressed in macrophages co-cultured with HCC-exo carrying oe-DLX6-AS1 (Fig. 6c). Therefore, a targeting relation between DLX6-AS1 and miR-15a-5p was speculated. Importantly, informatics tools (microRNA.org-Targets and Expression software) searched out the potential binding sites between DLX6-AS1 and miR-15a-5p (Fig. 6d) and dual luciferase reporter test further verified their targeting relation, as evidenced by the experiment, cells co-transfected with DLX6-AS1-WT and miR-15a-5p mimic had weakened luciferase activity (Fig. 6e). RIP assay was performed to further confirm the endogenous binding of miR-15a-5p and DLX6-AS1. It was found that in the miR-15a-5p up-regulation model, the immunoprecipitation containing anti-Ago2 antibody indicated that there was a strong binding between DLX6-AS1 and miR-15a-5p (Fig. 6f). Additionally, this binding relationship was further confirmed using RNA pull-down assay (Fig. 6g). Next, miR-15a-5p inhibition was conducted in macrophages (Fig. 7a). More importantly, inhibiting miR15a-5p facilitated M2 polarization (Fig. 7b, c; Supplementary Figure), thereby promoting migration, invasion and EMT of SMMC-7721 and HepG2 cells (Fig. 7d-f).

**Fig. 6:** DLX6-AS1 interacts with miR-15a-5p. **a**. RT-qPCR detection of miR-15a-5p expression in cancer tissues and normal tissues; **b**. RT-qPCR detection of miR-15a-5p expression in cancer cells and normal liver cells; **c**. RT-qPCR detection of miR-15a-5p expression in macrophages after co-culture with HCC-exo delivering oe-DLX6-AS1; **d**. Prediction of the potential binding sites of DLX6-AS1 and miR-15a-5p through bioinformatics websites; **e**. Verification of the targeting relationship between DLX6-AS1 and miR-15a-5p through dual luciferase reporter experiment; **f**. RIP detection of the binding relationship between DLX6-AS1 and miR-15a-5p; **g**. RNA pull-down detection of the binding relationship between DLX6-AS1 and miR-15a-5p; data were expressed as mean ± standard deviation (repetition = 3) and evaluated by One-way AVONA and Tukey’s test. * *P* < 0.05 compared with the oe-NC-exo group

**Fig. 7:** Down-regulating miR-15a-5p promotes M2 macrophage polarization and HCC cell migration, invasion and EMT. **a**. RT-qPCR detection of miR-15a-5p expression in macrophages after down-regulating miR-15a-5p; **b**. RT-qPCR detection of M2 macrophages markers (CD206, CD163, CCL17 and CCL18) after down-regulating miR-15a-5p; **c**. RT-qPCR detection of M1 macrophages markers (TNF-α, IL-6 and TGF-β) after down-regulating miR-15a-5p; **d**. Transwell assay tested the migration and invasion of SMMC-7721 cells after co-culture with macrophages inhibiting miR-15a-5p; **e**. Transwell assay tested the migration and invasion of HepG2 cells after co-culture with macrophages inhibiting miR-15a-5p; **f**. E-cadherin, N-cadherin, vimentin and MMP7 expression in SMMC-7721 and HepG2 cells after co-culture with macrophages inhibiting miR-15a-5p by qPCR; data were expressed as mean ± standard deviation (repetition = 3) and evaluated by One-way AVONA and Tukey’s test. % *P* < 0.05 compared with the NC-inhibitor group; + *P* < 0.05 compared with the NC-inhibitor + M group

### DLX6-AS1 mediates miR-15a-5p to target CXCL17 to drive migration, invasion and EMT in HCC

CXCL17, an overexpressed gene in HCC is associated with poor prognosis [17]. The same trend of CXCL17 was found in clinical cancer tissues (Fig. 8a) and in SMMC-7721 and HepG2 cell lines (Fig. 8b). In addition, inhibiting miR-15a-5p could elevate CXCL17 level in macrophages (Fig. 8c). Moreover, the potential binding sites between CXCL17 and miR-15a-5p were found through the informatics tools (microRNA.org-Targets and Expression software) (Fig. 8d) and the luciferase reporter gene assay displayed that co-transfection of CXCL17-WT and miR-15a-5p mimic repressed cell luciferase activity (Fig. 8e). Given the fact that CXCL17 triggered the polarization of monocytes into M2 macrophages [26], it was speculated to take part in DLX6-AS1/miR-15a-5p axis-mediated polarization of M2 macrophages in HCC metastasis. Next, in response to CXCL17 silencing in macrophages (Fig. 9a), M2 macrophages were polarized (Fig. 9b, c; Supplementary figure). After co-culturing with CXCL17-silenced macrophages, the migration and invasion abilities of HCC cells were weakened (Fig. 9d, e). EMT was also suppressed by CXCL17-silenced macrophages (Fig. 9f). Subsequently, we co-cultured CXCL17-inhibiting macrophages with HCC-exo carrying oe-DLX6-AS1, and tested the transfection efficiency by RT-qPCR (Fig. 10a). We found that after the co-culture, the polarization of M2 macrophages was inhibited (Fig. 10b, c, Supplementary Figure) and the migration and invasion and EMT abilities of SMMC-7721 and HepG2 cells (Fig. 10d-g). These results concluded that CXCL17, as a target gene of miR-15a-5p, was involved in the process of DLX6-AS1/miR-15a-5p axis-induced polarization of M2 macrophages to promote HCC migration, invasion and EMT.

**Fig. 8:** DLX6-AS1 mediates miR-15a-5p to target CXCL17 to drive migration, invasion and EMT in HCC. **a**. RT-qPCR analysis of CXCL17 expression in clinical tissues; **b**. RT-qPCR and Western blot analysis of CXCL17 expression in cancer cells and normal liver cells; **c**. RT-qPCR and Western blot analysis of CXCL17 expression in macrophages after down-regulating miR-15a-5p; **d**. Prediction of the potential binding site of miR-15a-5p and CXCL17 through bioinformatics websites; **e**. Verification of the targeting relationship between miR-15a-5p and CXCL17 through dual luciferase reporter experiment; data were expressed as mean ± standard deviation (repetition = 3) and evaluated by One-way AVONA and Tukey’s test. $ *P* < 0.05 compared with HL-7702 cells; & *P* < 0.05 compared with the NC-inhibitor group

**Fig. 9:** DLX6-AS1 mediates miR-15a-5p to target CXCL17 to drive migration, invasion and EMT in HCC. **a**. RT-qPCR and Western blot analysis of CXCL17 expression in macrophages after silencing CXCL17; **b**. RT-qPCR detection of M2 macrophages markers (CD206, CD163, CCL17 and CCL18) after silencing CXCL17; **c**. RT-qPCR detection of M1 macrophages markers (TNF-α, IL-6 and TGF-β) after silencing CXCL17;**d**. Transwell assay tested the migration and invasion of SMMC-7721 cells after co-culture with macrophages inhibiting CXCL17; **e**. Transwell assay tested the migration and invasion of HepG2 cells after co-culture with macrophages inhibiting CXCL17; **f**. E-cadherin, N-cadherin, vimentin and MMP7 mRNA expression in SMMC-7721 and HepG2 cells after co-culture with macrophages inhibiting CXCL17; data were expressed as mean ± standard deviation (repetition = 3) and evaluated by One-way AVONA and Tukey’s test; % *P* < 0.05 compared with the si-NC group; + *P* < 0.05 compared with the si-NC + M group

**Fig. 10:** DLX6-AS1 mediates miR-15a-5p to target CXCL17 to drive migration, invasion and EMT in HCC. **a**. RT-qPCR analysis of CXCL17 expression in macrophages; **b**. RT-qPCR detection of M2 macrophages markers (CD206, CD163, CCL17 and CCL18); **c**. RT-qPCR detection of M1 macrophages markers (TNF-α, IL-6 and TGF-β); **d**. Transwell assay tested the migration and invasion of SMMC-7721 cells; **e**. Transwell assay tested the migration and invasion of HepG2 cells; **f/g**. E-cadherin, N-cadherin, vimentin and MMP7 mRNA expression in SMMC-7721 and HepG2 cells; data were expressed as mean ± standard deviation (repetition = 3) and evaluated by One-way AVONA and Tukey’s test. ^ *P* < 0.05 compared with the oe-DLX6-AS1-exo + si-NC group; + *P* < 0.05 compared with theoe-DLX6-AS1-exo + si-NC+ M group

### DLX6-AS1 from HCC-exo promotes lung metastasis by inducing M2 macrophage polarization in mice with HCC

Next, we further explored whether HCC-exo DLX6-AS1 could also induce M2 macrophage polarization to promote HCC metastasis in vivo. The macrophages were treated with PBS or co-cultured with HCC-exo transfected with oe-NC/DLX6-AS1. Subsequently, the treated macrophages, together with SMMC-7721 cells were in situ injected into the right liver lobe. After 3 weeks, the mice were euthanized and the lungs were collected. After HE staining, metastases were mostly distributed in the peripheral lungs, mainly micrometastases in the interstitium and parenchyma; some intravascular tumor thrombi can be seen, and micrometastases were mostly composed of dozens of cancer cells; inflammatory cells were gathered, with lightly stained nucleus and less cytoplasm (Fig. 11a). The number of tumor lung metastases was calculated, and showed to increase after HCC-exo treatment while further enhanced by restored DLX6-AS1 from HCC-exo (Fig. 11b) In summary, HCC-exo DLX6-AS1 induced M2 macrophage polarization in vivo to promote lung metastasis of HCC cells.

**Fig. 11:** DLX6-AS1 from HCC-exo promotes lung metastasis by inducing M2 macrophages in mice with HCC. **a**. H&E-stained tumor tissues (200 ×); **b**. Number of metastatic hepatic nodules; data were as the mean ± standard deviation (mice = 6/group) and evaluated by One-way AVONA and Tukey’s test

## Discussion

Liver cancer is a non-communicable disease that requires coordinated global action to control [37]. In this research, we testified the actual actions of DLX6-AS1 from HCC-exo in the process of HCC cell invasion, migration and EMT. Through statistical analysis, HCC-exo were discovered to induce M2 macrophage polarization, thereafter to activate the metastatic activities of HCC cells. Then, DLX6-AS1 was examined to be overexpressed in HCC and then triggered cells to migrate and invade and accelerated EMT. In combination, HCC-exo could deliver DLX6-AS1 to promote lung metastasis in vivo through stimulating M2 macrophage polarization. Finally, DLX6-AS1 could interact with miR-15a-5p to target CXCL17, and then regulate migration, invasion and EMT in HCC.

Some reports have investigated the functions of HCC-exo in human cancers. For instance, promoted migration, invasion and EMT, as well as reduced E-cadherin and elevated Vimentin levels are detected in HCC cells that have been co-cultured with HCC-exo and in vivo lung metastasis is enhanced by HCC-exo treatment [38]. Another research summarizes intriguingly that exosomes from high-metastatic HCC cells are aggressive to promote HCC cell migration and can even convert the low-metastatic potential of HCC cells to a high level [39]. Also, invasive HCC-exo have been studied to eliminate drug efficacy and then facilitate HCC cellular growth [40]. Exosomes secreted by high-metastatic HCC cells are the driving actor for the migratory and invasive behaviors of low metastatic HCC cells, as well for EMT process (increased vimentin and reduced E-cadherin) [41]. Statistical analysis by a late study has profiled that HCC-exo could motivate M2 macrophage polarization to push forward the process of HCC [9]. M2 macrophages are multifunctional to incur HCC cell migration and metastasis [42]. Exactly, extracellular ubiquitin-induced M2 macrophage polarization has been known to provoke lung metastasis of HCC cells [43]. Also, tumor cells-derived Wnt ligands-stimulated M2 macrophage polarization acts as an indirect actor for the migration and metastasis of HCC cells [44].

LncRNAs have been extensively discussed to modify M1/M2 macrophage polarization and to mediate metastatic behaviors of liver cancer cells [45, 46]. Though the regulatory effect of DLX6-AS1 on M1/M2 macrophage polarization has not been discussed yet, its actions in cancer progression has been explored in reported studies. As mentioned before, DLX6-AS1 is overexpressed in HCC and its depletion would depress the stemness of liver cancer stem cells [12]. DLX6-AS1 silencing in HCC cells could disrupt the cellular migration and invasion [13, 33]. Therefore, DLX6-AS1 is further supported as the pro-tumor actor in HCC.

LncRNAs often function in diseases through modulating miRNAs. At present, the concrete actions of miR-15a-5p in liver cancer have been argued. For instance, reduced miR-15a-5p has been measured in HCC which is related to cellular growth [14, 15]. and miR-15a-5p inhibition in HCC is the stimuli for the metastasis of malignant cells [47]. Also, the elevated level of miR-15a-5p blockades the way of EMT in prostate cancer [48], as well as the migration and invasion of lung cancer cells [49]. It is noted that the elevated miR-15a-5p in chronic myeloid leukemia exerts to repress cell metastasis via targeting CXCL10 [16]. In our study, CXCL17 was confirmed as a target of miR-15a-5p which was involved in HCC process. As reported previously, CXCL17 is the exact up-regulated actor in HCC, whose restoration enhances invasion and migration of HCC cells while its reduction causes the opposite reactions [18]. In fact, enhanced level of CXCL17 is connected with disease progression in lung/hepatic cancer [50] and it is also the inducer of lung adenocarcinoma spine metastasis [51].

## Conclusion

Collectively, it was drawn from this research that HCC-exo delivered DLX6-AS1 to macrophages to stimulate M2 macrophage polarization, thus to irritate the invasion, migration and EMT of HCC cells in vitro and lung metastasis in vivo, which was related to the regulation of miR-15a-5p/CXCL17 axis. A novel pathway has been paved for understanding the molecular mechanism in HCC. Scientific confirmation and development are required for this research in the future in a larger cohort.

## Supplementary Information

**Additional file 1: Supplementary Figure.** Flow cytometry detection of M2 macrophage surface marker CD206. Data were expressed as mean ± standard deviation (mice = 6/group) and evaluated by One-way AVONA and Tukey’s test. * *P* < 0.05.

## Data Availability

Not applicable.

## Abbreviations

HCC: Hepatocellular carcinoma
HCC-exo: Hepatocellular carcinoma cells-secreted exosomes
CXCL17: C-X-C motif chemokine ligand 17
lncRNA: Long non-coding RNA
miRNAs: MicroRNAs
CXCL10: C-X-C motif chemokine ligand 10
ANOVA: Analysis of variance
TNF-α: Tumor necrosis factor-α
IL: Interleukin
TGF-β: Transforming growth factor β
